The article "An Optimization Analysis Model of Tourism Specialized Villages Based on Neural Network and System Dynamics" was published in 2022. Journal: Comput Intell Neurosci.

# An Optimization Analysis Model of Tourism Specialized Villages Based on Neural Network and System Dynamics

**DOI:** 10.1155/2022/2207814

**Published:** 2022-05-17

**Authors:** Wei Wang, Shiqi Yu, Suiying Cheng, Kaixia Liu, Shuang Jia

**Affiliations:** ^1^School of Culture Industry and Tourism Management, Henan University, Kaifeng 475001, Henan, China; ^2^College of Geography and Environmental Science, Henan University, Kaifeng 475001, Henan, China; ^3^Facultad de Ciencias Jurídicas y de la Empresa, Universidad Católica San Antonio, Murcia 30100, Spain

## Abstract

With the rapid development of tourism, professional tourism villages emerge one after another, which has become the focus of the tourism industry. At present, there are some problems in tourism professional villages, such as imperfect management and inaccurate prediction of future development, which affect the rational allocation of tourism resources. In order to improve the distribution of tourism resources and better predict the development of tourism professional villages, it is necessary to make comprehensive judgment and analysis, especially the analysis of indicators such as the prediction and development judgment of tourism professional villages. This paper discusses the optimization analysis of the agglomeration of tourism specialized villages by backpropagation (BP) neural network and system dynamics model, analyzes the system structure of the agglomeration factors of tourism specialized villages, and promotes the intelligent integration of the agglomeration factors. The development of clusters of professional villages promotes data integration among resources, economy, society, and other elements and presents the characteristics of big data. As the level of concentration of professional villages increases, the complexity of the associated factors also increases, which increases the difficulty and effectiveness of tourism analysis. In view of this situation, taking mountain tourism as the research object, this paper proposes an improved system dynamics model based on BP, extracts features from cross factor (resource, economic, and social) data, and optimizes the relationship between professional village agglomeration and various factors. The MATLAB simulation results show that based on the improved system dynamics analysis, the simplification rate of (resources, economy, and society) data can be controlled at more than 24%, the degree of agglomeration is more than 95%, and the construction time of the relationship map of related factors is less than 40 s. Therefore, the analysis method proposed in this paper is suitable for the calculation of the agglomeration of tourism professional villages in the mountain area and can meet the needs of the development of tourism professional villages in the mountain area.

## 1. Introduction

Different from other tourism projects, tourism professional village is a tourism project integrating mountain tourism and professional tourism. The project can not only optimize the existing tourism industry structure but also optimize the future development. Tourism professional village is more professional and develops rapidly. It is the main development project in China, so it has very important practical significance. The research of scholars at home and abroad mainly stays at the theoretical level and lacks specific practical operation. At the same time, the research focuses on qualitative aspects and lacks comprehensive analysis. Therefore, a comprehensive analysis of tourism professional villages is an urgent problem to be solved. Domestic research on tourism professional villages is mainly theoretical comparison, or copying foreign models, lacking a way suitable for domestic needs. Therefore, the research on tourism professional village combined with local characteristics has important theoretical significance.

System dynamics have been developed over a long period of time and have been used extensively in many areas. They have been applied in economic and other areas in depth, but there is little research on tourism in mountainous regions. The dynamics of the system can efficiently integrate the attribute data of degree of professional village agglomeration. Combined with the system dynamics theory, the development of tourism specialized villages is analyzed in the study of Arif [1]. According to the survey data of tourism professional villages, the development direction is analyzed. At the same time, combined with the existing conditions of tourism specialized villages (infrastructure, market share, and brand effect) in the study of Benaraba [2], this paper makes a multi-angle study. Under the dual effects of neural network and system dynamics, the development direction of tourism specialized villages is accurately judged. Some scholars believe that the study of tourism specialized villages is difficult, which is mainly reflected in two aspects. On the one hand, the study of tourism specialized villages is affected by many factors, and the calculation process is complicated in the study of Deng et al. [3]. On the other hand, the analysis process of tourism specialized villages is tedious, and the general analysis methods cannot be accurately analyzed.

Compared with foreign scholars, domestic scholars pay more attention to theoretical research and lack of practical case analysis. At the same time, when domestic scholars introduce foreign research content, they find that they cannot copy it, so they need to verify relevant cases. Therefore, this paper takes the economic dynamics, resource information, social structure, and other related fields as the scope, constructs the system dynamics model between the agglomeration of specialized villages and related factors, analyzes the effectiveness, accuracy, and calculation time of the model, and provides data and case support for the adjustment and management of the agglomeration of specialized villages.

## 2. Literature Review

There are many studies on system dynamics or BP neural networks, but they mainly focus on tourism management and lack of research on the tourism agglomeration of mountain villages. Some researchers believe that mountain tourism will be the main direction of tourism development in the future, while scattered tourism research cannot find the development law [5]. Some scholars also believe that the key to mountain village tourism is to analyze the professional villages, analyze the areas where the professional villages gather, and find out the differences [6]. Some scholars believe that the personalization of mountain village tourism is obvious, and the reasons for its agglomeration should be analyzed [7]. Some scholars believe that applying the theory of system dynamics to mountain village tourism can find out the characteristics of mountain village tourism through the analysis of the driving factors of tourism. Some researchers also believe that the dynamics of the system have its own limitations, making it impossible to conduct a thorough analysis of the combined professional villages [8]. They should be improved and the method of cluster analysis should be introduced appropriately. To sum up, scholars at home and abroad believe that mountain village tourism is the future development direction and suggest introducing BP neural network method for analysis [9]. Domestic mountain village tourism is in its early stages and lacks practical case analysis, while foreign case studies cannot be copied. Therefore, we should learn from foreign experience and make a comprehensive analysis of mountain village tourism [10]. On this basis, this paper improves the system dynamics and applies this method to the tourism analysis of professional villages in the mountainous areas in order to accurately judge the agglomeration of professional villages.

## 3. Research Mode

### 3.1. The Analysis and Description of the Agglomeration Relationship of Vocational Tourism Villages in the Mountainous Region

The essence of agglomeration is the association based on the customer relationship database (CRD) [11]. The data fusion of related fields involves the nodes of multifield data and the relationship lines of various types of related factors and forms the dynamic diagram of complex system, which is also the mapping of the agglomeration relationship of real professional villages [12]. Compared to the merging of data from other related fields, the relationship between the factors influencing the agglomeration of professional villages is more complex [13], and unstructured data represent more than 80%, and the complex merging of unstructured and structured data further increases the construction of the map. Therefore, it is necessary to conduct mathematical analysis on the agglomeration relationship of specialized villages and lay the foundation for later quantitative analysis [14].

### 3.2. Analysis of System Dynamics

There are two difficult problems in cross domain data fusion. (1) Massive unstructured cluster data, partial semi-structured cluster data, and low value cluster data increase the processing capacity of fusion cluster data [15]. (2) Multisource dynamic cluster data increase the complexity of fusion systems. The above two challenges reduce the accuracy and efficiency of system dynamics analysis [16]. System dynamics should analyze the influencing factors of tourism specialized villages, such as economic factors, social factors, and tourism specialized villages themselves [17]. Among the nodes in system dynamics analysis, BP neural network is integrated into the model construction, which can not only judge the subordinate relationship between different nodes but also judge the attributes between different nodes. BP neural network can also eliminate the nodes in the system, bring the nodes that meet the threshold into the system dynamics, reduce the number of useless nodes, and improve the analysis speed of relevant data.

### 3.3. Description of the Aggregated Data Stream

In order to analyze more precisely the fusion of agglomeration data and to construct an objective relationship diagram of the agglomeration of the specialized village, it is necessary to describe the flow of agglomeration data. At present, there are many analysis methods for clustered data stream, but it is difficult to carry out comprehensive analysis, and it is also difficult to extract feature data from the data collected by Python, which increases the calculated amount of clustered data.

(1) It is assumed that the research results index of tourism specialized villages are as follows: 1) *xi* is the present situation of tourism specialized villages agglomeration; 2) *xj* is the resource concentration degree of tourism specialized villages. Among them, the data set of resources, economy, and social structure are *C* = {*c*_1_, *c*_2_,…, *c*_*i*_}. Then, the relationship between aggregate data and system dynamics is
  (1) $$\begin{array}{c} c_{i}\overset{=}{\underset{\underset{\text{Results feedback}}{\leftarrow }}{⟶}}\bar{\sum_{i,j,k}^{n}x_{i}+x_{j}}, \end{array}$$
where *I* and *j* belong to natural numbers.
(2) Suppose that the cluster data information is *key*, *I* is the industry of the cluster data source (monuments = 1, nature = 2, and humanities = 3) [18], *j* is the type of cluster data (structured cluster data = 1, semi-structured = 2, and unstructured = 3), and *k* is the processing method of cluster data (industry standard = 1, relevant industry standard = 2, and this industry standard = 3); then, *I* is described as *c*_*i*_^*I*,*j*,*k*^, *I*, *j*, *k* ∈ (1,2,….., *n*), and *n* is a nonzero natural number.
(3) The fusion function *φ*(*x*) is used to calculate the fusion degree [19].
(4) The agglomeration data of different fields should be based on the agglomeration of specialized villages. The construction time *T* of the system dynamics model [20], the calculation effect *θ*, and the simplification rate of the agglomeration data *w*_*I*_ collected by Python should be calculated. The specific formula is as follows:
  (2) $$\begin{array}{c} \sum w_{I}\%=\frac{H\cdot G_{Ij}}{G_{I}+G_{j}}\cdot \frac{100}{n}, \end{array}$$
where *G*_*Ij*_ is the number of *I* industry information of *j* cluster data, *G*_*I*_ is the total amount of *I* industry information in the cluster database of suburban mountain tourism professional village, *G*_*j*_ is the total amount of *j* cluster data, and *w*_*i*_ is the simplification degree of *I* tourism professional village related information.
(5) In order to ensure that the calculated agglomeration data meet the development standards of tourism professional villages in the mountain area [21], it is necessary to set the weight *ω* and threshold of the fusion agglomeration data *ρ* to get the fusion agglomeration data $\hat{\underset{x⟶\infty }{\lim}f\left(x\right)}$.
(6) In order to simplify Python's collection of tourism village cluster data, k-means clustering algorithm (k-means) processing method is used to limit Python cluster data, and the initial clustering range is obtained by $\tilde{\left|S\right|=\sum_{i=0}^{n}c_{i}}$.

### 3.4. Building a Model for Optimizing the Agglomeration of the Specialized Village of Tourism Based on the Neural Network and the Dynamics of the System

First, the standardized processing of relevant research data is done. Before building the cluster analysis of professional tourist villages in the mountain area, it is necessary to simplify the cross domain cluster data and obtain the characteristic cluster data. In this article, we use the method of system dynamics to judge the importance depending on the neural network. Only when the original baseline is 50% [22], can it be selected as original agglomeration data. Assuming that the initial value of agglomeration data is *V*_*I*_, whether it needs to improve its own value, that is, the transformation from *V*_*I*_ to *V*_*I*+_ 1, should be calculated by the following formula:

(3) $$\begin{array}{c} P\left(V\right)\left\{\begin{array}{c} \text{Raw}\underset{x⟶\infty }{\lim}0∼0.5,f\left(I\right)⟶f\left(I\right),\text{ and }f\left(I\right)=0,\\ \text{Raw Between }0.5∼1,\text{exp}\left[f\left(I\right)-\frac{f\left(I+1\right)}{V_{I}}\right]\neq 0,\text{ and }f\left(I+1\right)=V_{I+1},\\ \text{Raw}=1,\text{ or }0,f\left(I\right)⟶f\left(I\right),\text{ and }f\left(I\right)=0,\text{ or }1. \end{array}\right. \end{array}$$

Among them, exp () is the judgment function of agglomeration, which is the basis to improve the degree of agglomeration; *P*(*V*) is the calculation function of the probability of agglomeration, which is mainly based on whether the importance of agglomeration data will be improved under different conditions. It can be seen from the above analysis that when the initial agglomeration degree of the agglomeration data is at 0 ~ 1/2 [23], the agglomeration data are eliminated; when the initial agglomeration degree of the agglomeration data is at 1/2 ~ 1 [24], the agglomeration data are accepted by exp(), and the corresponding calculation is performed. According to the neural network, the improvement in the degree of agglomeration of agglomeration data is considered. Where data on the degree of initial agglomeration are used to calculate the degree of agglomeration, data on the degree of initial agglomeration should be maintained. Secondly, the analysis of influencing factors affects the development of tourism specialized villages. The relationship between society, resources, economy, and related factors of specialized village agglomeration is complex, which can be judged by partial fitting PC and overall fitting *P*_*M*_. Local fitting is divided into two parts: local fitting *P*_*C*1_ of cross domain agglomeration data and local fitting *P*_*C*2_ of relevant factors of specialized village agglomeration. The overall adjustment reflects the relationship between the interdomain agglomeration data and the relevant factors of the agglomeration specialized village [25], which is the final adjustment value to be achieved in building this model.

(4) $$\begin{array}{c} P_{c}\left\{\begin{array}{c} P_{c_{i}^{1,1,1}}\cup P_{c1}=P_{\text{c}2},\\ \frac{\varphi \left(x\right)\left[\left(P_{c1}-P_{\min}\right)+\left(P_{c2}-P_{\min}\right)\right]}{2\left(P_{c_{i}^{I,j,k}}-P_{\min}\right)}\cap P_{c1}\neq P_{c2}, \end{array}\right.\underset{\text{neural network}}{\underset{↽}{⇀}}, \end{array}$$

where *P*_*c*_*i*_^1,1,1^_ is the initial value; min[*P*_*m*_] and *P*_min_ is the minimum value of *P*_*C*_ and *P*_*M*_ agglomeration data; and *φ*(*x*) is the agglomeration degree function. Third, the accuracy analysis of the research on the development of tourism specialized villages is done [26]. The precision of the cluster analysis of tourism villages in the mountainous area is an important criterion for judging the advantages and disadvantages of the model. Taking system dynamics as the prototype, this paper judges the accuracy of the results, which involves three aspects: whether the calculated results are in line with different regional thresholds, the threshold of interregional system relationship, and the overall threshold of specialized village agglomeration. In the case of the initial precision requirements, the three aspects of the data adjustment are evaluated with precision to obtain the calculation precision of the relationship graph. The formula for calculating this is [27]

(5) $$\begin{array}{c} F\left(y\right)=\left\{\begin{array}{c} \left[\frac{F\left(y_{i}\right)}{n}\right]\underset{\text{neural network}}{⥂}\min\left[f\left(c_{i}^{1,1,1}\right)\right]∵\left[df\left(P_{c_{i}^{I,J,K}}\right)\right]\neq 0,\\ f\left(P_{c_{i}^{I,J,K}}\right)\underset{\text{neural network}}{⥄}1\exists \int_{I,j}^{n}\left(\sum_{I=1}^{n}\max\left(F\left(y_{i}\right)≐F\left(y_{i+1}\right)\right)∵\prod \underset{c⟶\infty }{\lim}\sqrt{i^{2}-4Ij}.\right. \end{array}\right. \end{array}$$

Among them, *F*(*y*) is the calculation result of economy, resources, and society, *f*(*P*_*c*_*i*_^*I*,*J*,*K*^_) is the calculation precision of agglomeration data, ∫_*I*,*j*_^*n*^(∑_*I*=1_^*n*^max(*F*(*y*_*i*_)≐*F*(*y*_*i*+1_)) is the maximum result in line with the calculation precision, *df*(*P*_*c*_*i*_^*I*,*J*,*K*^_) is the derivative of the final result, $\prod \underset{x⟶\infty }{\lim}\sqrt{i^{2}-4Ij}$ is the error function, and min[*f*(*c*_*i*_^1,1,1^)] is the initial minimum value [28]. Fourthly, in the study of tourism specialized villages, the role of neural network is combined with system dynamics model.

According to the above formula construction, the following calculation steps are carried out [29]:

1. Construct information set, *C* = {*c*_1_,*c*_2_,…, *c*_*i*_}. Python data with a degree of clustering less than 50% are deleted, and the threshold, weight, and accuracy threshold are defined.
2. The system dynamics method is used to assess the degree of agglomeration as a function of the neural network. If *f*(*I*)⟶*f*(*I*), the weight of the aggregation data is assigned to $\underset{i⟶\infty }{\lim}0$; otherwise, the weight is assigned.
3. The fitting values of *P*_*C*_ and *P*_*M*_ were calculated.
4. Python data adjustments are scanned, and MATLAB simulation analysis is performed in accordance with the 50 predefined iterations.
5. The measured values of system dynamics analysis are outputs.

## 4. Case Analysis Based on Neural Array and System Dynamics Model

Based on the improvement of the dynamics of the system, the verification of the model of agglomeration of professional tourist villages in the mountain area is conducted.

### 4.1. Description of Actual Situations

This paper takes baoduzhai Scenic Spot, the first scenic spot in Luanchuan County, as the research object, and the data collection time is from 1992 to 2020 [30]. Among them, the output precision of Xi, XJ, and XK is 0.1, and the initial value is 78%, the local threshold is 69%, and the number of iterations is 50. Python collected 131 data, accounting for 23.1% of resource data, 72.3% of social structure data [31], and 3.6% of the economy.

### 4.2. Streamlining Python Data

Using the neural network and the k-means grouping, the domain grouping data are simplified, as shown in Figure 1.

As shown in Figure 1, different treatments for the complexity of Python data are ideal, and they are all over 24%. Of these, the level of simplification of data from resource clusters is the highest, followed by data from economic clusters and data from social clusters. The reason for the above phenomenon is that the data of resource agglomeration are more repetitive and have a lower impact on the agglomeration of specialized villages [32]; therefore, the level of simplification is greater. Data on economic agglomerations are closely related to specialized village agglomerations but are also simplified by fixed interest rates and long-term economic policies. Although Python's search results in a surge in the amount of aggregated data, the social structure is relatively stable and has a great impact on the degree of agglomeration, so the simplification rate of complexity is only about 24%. In addition, the change trends of source data, social structure data, and economic data in Figure 1 are basically the same, which shows that the analysis results of the above three indicators by the framework model in this paper are ideal. At the same time, the economic data changes greatly, mainly because economic development is greatly affected by policies and regions.

### 4.3. The Degree of Merging and the Accuracy of the Calculation of Aggregated Data

Under the accuracy standard of 0.1, this paper analyzes the integration degree PC and the overall integration degree PM of the factors related to the agglomeration of specialized villages in the fields of economy, social structure, and resources. The specific outcomes are presented in Figure 2.

In the above analysis results, the highest degree of cross domain integration is due to the more dynamic factors related to the agglomeration of professional villages and the higher statistical difficulty of cross domain agglomeration data, but the overall integration degree is higher, which is higher than 95%, and the accuracy is >95%, so the overall accuracy calculation result is better [33]. The degree of data fusion is good, and only one inflection point appears in 44 iterations. The turning point of local data fusion in the initial stage of calculation is mainly due to the large amount of data in the initial stage and complex operation. Compared with local data fusion, global fusion has two turns, mainly in the initial stage, which is also due to the large amount and complexity of data in the initial stage.

### 4.4. The Generation Time of Analysis of Agglomeration Relationship of Professional Tourist Villages in the Mountain Region

The generation time of the relation graph involves the settlement of nodes, the relation between nodes, and the global generation time of the graph. Depending on the above three aspects, the following simulation results are achieved, as shown in Figures 3 and 4.

Through the above analysis, we can see that the time of resource, economic, and social structures of the BP neural network and system dynamic relationship is within 50 s, which is in line with the standard of professional village agglomeration optimization.

To sum up, this paper uses system dynamics and neural network to analyze tourism professional villages. The results have significant advantages in data fusion, calculation simplification, and calculation time, which meet the development requirements of tourism professional villages.

## 5. Conclusion

How to promote the rapid development of professional village agglomeration, cross domain data analysis, and data fusion in resources, economy, society, and other fields, to promote the degree of tourism professional village agglomeration, and to build a system dynamics model with high accuracy is an urgent problem to be solved. This paper uses the K-mean method and the BP neural network to build an analysis model of the agglomeration of specialized villages of tourism in mountainous areas based on the BP neural network and system dynamics. The simulation results show the following. (1) The data simplification degree of Python in different fields is more than 24%. (2) The overall integration degree is more than 95%, and the accuracy is more than 95%. (3) The processing time of the resource, social, economic, and other data in the BP neural network and system dynamics is less than 50 s. (4) The changes among economic, social, and data sources are relatively stable, and the test curve is relatively smooth, close to 100%. Therefore, the optimization method proposed in this paper has strong applicability and can meet the needs of the development of professional village agglomeration.

## Figures and Tables

**Figure 1:** Simplification of various Python data.

**Figure 2:** Calculation of cross domain merger, local merger, and global merger.

**Figure 3:** The operating time of the neural network and the dynamics of the system at each stage.

**Figure 4:** The effect of neural network generation and system dynamics at each stage. (a) Resources. (b) Economy. (c) Social conditions.

## Data Availability

The data used to support the findings of this study are included within the article.
